The article "Classification of Hepatocellular Carcinoma and Intrahepatic Cholangiocarcinoma Based on Radiomic Analysis" was published in 2022. Journal: Comput Math Methods Med.

# Classification of Hepatocellular Carcinoma and Intrahepatic Cholangiocarcinoma Based on Radiomic Analysis

**DOI:** 10.1155/2022/5334095

**Published:** 2022-02-21

**Authors:** Xiaoliang Xu, Yingfan Mao, Yanqiu Tang, Yang Liu, Cailin Xue, Qi Yue, Qiaoyu Liu, Jincheng Wang, Yin Yin

**Affiliations:** ^1^Department of Hepatobiliary Surgery, The Affiliated Drum Tower Hospital of Nanjing University Medical School, Nanjing, China; ^2^Department of Hepatobiliary Surgery of Drum Tower Clinical Medical College, Nanjing Medical University, Nanjing, China; ^3^Department of Radiology, The Second Affiliated Hospital of Nanjing Medical University, Nanjing, China; ^4^Preparatory School for Chinese Students to Japan, The Training Center of Ministry of Education for Studying Overseas, Changchun, China

## Abstract

**Introduction:**

Considering the narrow window of surgery, early diagnosis of liver cancer is still a fundamental issue to explore. Hepatocellular carcinoma (HCC) and intrahepatic cholangiocarcinoma (ICCA) are considered as two different types of liver cancer because of their distinct pathogenesis, pathological features, prognosis, and responses to adjuvant therapies. Qualitative analysis of image is not enough to make a discrimination of liver cancer, especially early-stage HCC or ICCA.

**Methods:**

This retrospective study developed a radiomic-based model in a training cohort of 122 patients. Radiomic features were extracted from computed tomography (CT) scans. Feature selection was operated with the least absolute shrinkage and operator (LASSO) logistic method. The support vector machine (SVM) was selected to build a model. An internal validation was conducted in 89 patients.

**Results:**

In the training set, the AUC of the evaluation of the radiomics was 0.855 higher than for radiologists at 0.689. In the valuation cohorts, the AUC of the evaluation was 0.847 and the validation was 0.659, which indicated that the established model has a significantly better performance in distinguishing the HCC from ICCA.

**Conclusion:**

We developed a radiomic diagnosis model based on CT image that can quickly distinguish HCC from ICCA, which may facilitate the differential diagnosis of HCC and ICCA in the future.

## 1. Introduction

According to the latest report of the International Agency for Research on Cancer, liver cancer is one of the most common digestive cancers. Primary liver cancer is the sixth most commonly occurring cancer and the third leading cause of cancer-related deaths worldwide, ranking fifth in incidence and fourth in mortality [1]. Despite the available treatment options, the incidence and mortality rates are nearly equal [2]. Surgery, with a narrow therapeutic window, remains the mainstay of liver cancer therapy for patients at early stage [3]. Thus, early diagnosis is still a fundamental issue to explore.

The article "Classification of Hepatocellular Carcinoma and Intrahepatic Cholangiocarcinoma Based on Radiomic Analysis" was published in 2022. Journal: Comput Math Methods Med.

The dominant histological types of primary liver cancer are hepatocellular carcinoma (HCC) and intrahepatic cholangiocarcinoma (ICCA), accounting for over 99% of primary liver cancer cases [4, 5]. Considering the clinical stages, patients with HCC and ICCA may be assigned to similar clinical managements [6]. However, HCC and ICCA are considered as completely different two types of liver cancer because of their distinct pathogenesis, pathological features, prognosis, and responses to adjuvant therapies [7]. Therefore, early discrimination of these two types of liver cancer contributes to designing personalized treatment strategies.

Computed tomography (CT), as a common type of imaging tool, plays a major part in diagnosis, staging, treatment, and follow-up of oncologic patients. During routine preoperative evaluation in a clinical setting, three-dimensional (3D) reconstruction of CT images helps formulate more reasonable surgical planning [8]. The contrast-enhanced CT provides higher resolution images and defines the nature of the lesion [9, 10]. However, the diagnostic accuracy is dependent on variations in radiologists' level of experience, resulting in frequent misdiagnosis [11]. Despite the development of modern imaging techniques, qualitative analysis of image is not enough to make a discrimination of liver cancer, especially early-stage HCC or ICCA, which have puzzled researchers for several years.

Radiomics, as a novel image processing technology, can automatically provide a large number of quantitative image features from medical images, which may be impossible for naked eyes to recognize [12, 13] These image features can also be combined with machine learning algorithms to make a prediction for diagnosis. Several studies have shown the outlook of prediction for cancer outcome [14]. The radiomic-based classifiers using routine magnetic resonance imaging (MRI) sequences in differentiation of peripheral schwannomas and neurofibromas showed higher area under the curve (AUC) values on the receiver operator characteristic (ROC) curve than expert human evaluators [15] and so was the random forest model based on CT radiomics [16]. Radiomics can significantly improve the accuracy and consistency of diagnosis. Unfortunately, very few studies have investigated the CT radiomic-based model to distinguish HCC and ICCA.

In this study, we established a support vector machine (SVM) based on radiomic features at noncontrast CT to train a discriminative model for HCC and ICCA at early stage. The diagnostic performance was also compared with experienced radiologists.

The article "Classification of Hepatocellular Carcinoma and Intrahepatic Cholangiocarcinoma Based on Radiomic Analysis" was published in 2022. Journal: Comput Math Methods Med.

## 2. Materials and Methods

### 2.1. Patients and Liver Pathological Diagnosis

The workflow is schematically depicted in Figure 1. All patients with pathologic results of liver cancer underwent noncontrast CT at our institution between August 2018 and November 2019. Here are the exclusion criteria for patient screening: (1) lack of abdominal noncontrast CT image at 1.5 mm thickness (*n* = 41), (2) poor image quality (*n* = 26), (3) an interval between pathological results and CT examination of more than 3 months (*n* = 11), (4) coinfection with virus such as HBV or HCV (*n* = 38), and (5) incomplete clinical data (*n* = 31).

We partitioned the whole cohort into two parts, 122 patients for training (from August 2018 to March 2019) and 89 patients for validation (from April 2019 to November 2019).

The clinical characteristics and the data of CT scan were obtained from medical records. Clinical data included age, sex, blood routine tests (red blood cell (RBC), white blood cell (WBC), platelet (PLT) count, and hemoglobin (Hb)), liver function examinations (ALT, aspartame aminotransferase (AST), alkaline phosphate (ALP), gluttony transpiration (GGT), lactate dehydrogenase (LDH), total bilirubin (TB), conjugated bilirubin (CB), albumin (ALB), globulin (GLOB), total bile acid (TBA), and leucine acrylamide (LAP)), lipid metabolism tests (total cholesterol (TC), high density lipoprotein cholesterol (HDL-C), low density lipoprotein cholesterol (LDL-C), apolipoprotein A1 (Apo A1), and apolipoprotein B (Apo B)), C-reactive protein (CRP), and blood coagulation function (prothrombin time (PT) and international normalized ratio (INR)).

The histopathological analysis of the liver was made by two pathologists with over 5-year working experience. And the pathologists were blinded to the clinical information.

### 2.2. CT Image Acquisition and Evaluation

All patients received the examination with the same CT scanner in supine position (LightSpeed, VCT, or Discovery HD 750, GE Healthcare, US). The CT scanner parameters are listed as follows: tube voltage 120 kVp, tube current 250–350 mA, collimating slice thickness 5 mm, reconstruction slice thickness 1.25 mm, slice interval 5 mm, rotation time 0.6 s, helical pitch 1.375, the field of view between 35 and 40 cm, and matrix 512 × 512. The image was reconstructed using a standard algorithm. The CT images were reviewed by two independent radiologists. The radiologists were aware of the diagnostic criteria and blinded to the clinical radiological details. Any differences were resolved through discussion.

### 2.3. The Establishment of Radiomic Model in the Training Cohort

Regions of interest (ROIs) were selected in the liver of all patients by two radiologists using 3D slicer (version 4.8.0; http://www.slicer.org) [17]. The ROIs were manually segmented along the tumor contour on each transverse section. Image preprocessing and feature extraction were performed by Pyradiomics package (http://www.radiomics.io/pyradiomics.html). The voxel spacing was standardized with the size of 1 × 1 × 1 mm. The voxel intensity values were discretized with a bin width of 25 HU to reduce the interference of image noise and normalize intensities [18]. Eight hundred forty-one radiomic features (13 shape statistics, 18 first-order statistics, 74 textural features, and 736 wavelet-based transformations) were extracted from each ROI (Table 1).

The article "Classification of Hepatocellular Carcinoma and Intrahepatic Cholangiocarcinoma Based on Radiomic Analysis" was published in 2022. Journal: Comput Math Methods Med.

The intra- and interobserver reliability for each radiomic feature was calculated by using intraclass correlation coefficient (ICC). Radiomic features with both intra- and interobserver ICC greater than 0.8 were selected for subsequent analysis. The least absolute shrinkage and selection operator (LASSO) logistic regression algorithm [19], along with penalty parameter tuning conducted by 10-fold cross-validation, was performed to select cirrhosis-related features (with nonzero coefficients).

### 2.4. Statistical Analysis

Categorical and continuous variables were compared by *χ*^2^ test and Student *t* test, respectively. The R package “e1071” was used to perform the SVM, and “glmnet” was used for LASSO regression on R software (version 3.6.1, http://www.r-project.org). The diagnostic performance of established models was evaluated by the ROC curve and area under the curve (AUC) value. The DeLong test was used to compare AUC values. Calibration curves were plotted via bootstrapping with 1000 resamples, accompanied by the Hosmer-Lemeshow test, to evaluate the calibration of the established model. The decision curve analysis (DCA) was used to calculate the net benefit from the use of established models. *P* < 0.05 was considered statistically significant.

## 3. Results

### 3.1. Baseline Characteristics

The clinical characteristics are shown in Table 2. There was no significant difference in age, sex, AFP, CEA, CA199 between the training, and validation cohorts.

### 3.2. Radiomic Analysis

Of 841 extracted features, 76 features (8 first-order statistics, 21 textural features, and 56 wavelet-based transformations) with high reproducibility were selected for subsequent analysis. 43 independent significant features were identified by the LASSO logistic regression model (Figure 2). A radiomic model was constructed using SVM algorithm, of which the type is eps-regression. The kernel function is radial-based and the number of support vectors is 73.

The article "Classification of Hepatocellular Carcinoma and Intrahepatic Cholangiocarcinoma Based on Radiomic Analysis" was published in 2022. Journal: Comput Math Methods Med.

### 3.3. Model Establishment and Validation

The ROC analysis is shown in Figure 3 and the summary of the model is shown in Table 3. In the training set, the AUC of the evaluation of the radiomics was 0.855 higher than for radiologists at 0.689. In the validation cohorts, the AUC of the radiomics model was 0.847 and the radiologic evaluation was 0.659, which indicated that the radiomics model have a significant benefit in distinguish the HCC form ICCA. The calibration of the training set model shows that the models established have a great agreement with the actual result and preside results. Besides, the curve of the validation cohorts shows the same results. The Hosmer-Lemeshow test yielded *P* values of 0.056 and 0.217 in the training and validation cohort, indicating no departure from the good fit.

The DCA is shown in Figure 4. Compared with scenarios in which no prediction model would be used (i.e., treat-all or treat-none scheme), the radiomic model can provide better net benefit in distinguishing the HCC from ICCA than radiologic evaluation for threshold probabilities of more than 20% in the training and validation cohorts.

## 4. Discussion

This is a brand new study for making a discrimination analysis for HCC and ICCA by establishing a radiomic-based classification model at noncontrast CT which showed higher efficacy than experienced radiologists. There are 43 selected radiomic features integrated in the model, and the great diagnostic performance was achieved.

HCC and ICCA are classified into liver cancer in the clinical classification but completely different in initiation and progression. First, viral infections, alcoholism, and fatty liver are leading risk factors for HCC, as primary sclerosing cholangitis, bile duct cyst, and hepatolithiasis are for ICCA. Second, HCC and ICCA originate from completely different cell population. It is generally believed that HCC is a highly aggressive epithelial tumor originating both from mature hepatocytes and stem cells [20]. However, ICCA is likely to arise from cholangiocytes or the epithelial cells lining the biliary tree [21]. Third, although surgical resection is the only preferred therapeutic option for both two cancers at early stage, the nonoperative treatment is significantly divergent [22]. Thus, early discrimination is of great value to cancer patients.

Unfortunately, the discrimination owes a major debt to image. The ability of radiologists plays major roles in that. Imaging examination mainly distinguishes them according to the difference of blood supply. The typical hepatocellular carcinoma has an abundant blood supply, which can facilitate the presence of nonrim-like enhancement of an observation in the arterial phase and the wash out in the venous phase [23]. Meanwhile, the hypovascular intrahepatic cholangiocarcinoma frequently results in insufficient enhancement of arterial phase [24]. But when it comes to nontypical HCC, it is difficult to identify HCC from ICCA [25]. The gold standard diagnostic test for liver cancer is the pathology, which need paracentesis or surgery. The selection of cancer diagnostics and treatments may delay for quite a long time. Therefore, it is necessary to find a more reliable, efficient, and user-friendly method to distinguish them.

The article "Classification of Hepatocellular Carcinoma and Intrahepatic Cholangiocarcinoma Based on Radiomic Analysis" was published in 2022. Journal: Comput Math Methods Med.

The contrast-enhanced CT or MRI, which can provide more information than noncontrast CT, was suggested by guidelines for patients with liver mass. However, many patients in China only accept noncontrast CT examinations because of limited cost-effectiveness (mainly attributed to price and waiting time). CT scan is one of the most economical, noninvasive, and convenient examination approaches along the presurgical evaluation and postoperative follow-up [26]. The radiomic approach relies on highly informative image data. Indeed, this is exactly why we selected radiomic analysis based on CT data. Researchers have determined the ability of MR perfusion-based radiomics to discriminate pseudoprogression from progressive disease in glioblastoma patients [27] and the normal tissue (glandular) from benign and malignant tumors in patients with breast mass [28].

There have been many liver cancer studies based on radiomics. However, these studies focused on the distinguishment of microvasculature and prediction of prognosis while may not meet the requirements for clinical application [29]. In this study, we established the model by analyzing the image features of patients and selected the features related to the pathological types of patients through logistic regression analysis. By analyzing the CT image features of the training cohort, we selected the image features with high correlation with patient diagnosis as factors of the radiomic model. To further verify the diagnostic validity of the data model, we validated this in the validation cohort. It is promising that the model we established has higher accuracy than experienced clinical radiologist. A stable radiomic-based model may play an important role in a regional hospital lack of experienced radiologists.

Meanwhile, some limitations pertain to our study. First, it is a retrospective study with some considerable risk of bias in the data-driven procedure. Second, the established model was based on a single center. Larger, multicenter cohort study analyses are needed to validate such model. Third, biochemical markers significantly contirbute to liver cancer-related studies, and this study did not involve biochemical markers into the established model. The analysis combining biochemical indicators and image features should be considered in the subsequent studies.

The article "Classification of Hepatocellular Carcinoma and Intrahepatic Cholangiocarcinoma Based on Radiomic Analysis" was published in 2022. Journal: Comput Math Methods Med.

## 5. Conclusion

In summary, we developed a radiomic diagnosis model based on CT image that can quickly distinguish HCC from ICCA, which may facilitate the differential diagnosis of HCC and ICCA in the future.

## Figures and Tables

**Figure 1:** The flow chart of the patients' inclusion.

**Figure 2:** Selection of radiomic features by the least absolute shrinkage and selection operator (LASSO) logistic regression. (a) Optimal *λ* value was determined by the LASSO model using 10-fold cross-validation via minimum criteria. The misclassification error curves were plotted versus log (*λ*). Dotted vertical lines were drawn at the optimal values by using the minimum criteria and the 1 standard error of the minimum criteria (the 1 –standard error criteria). The optimal *λ* value of 0.0442 was chosen.

**Figure 3:** The ROC and calibration curves of the radiomic model. Comparison of ROC curve between radiomic model and radiological evaluation in training (a) and validation (b) cohorts. The calibration curves of the radiomic model in the training (c) and validation (d) cohorts.

**Figure 4:** The decision curve analysis for radiomic model in the training (a) and validation (b) dataset. The net benefit was shown in the *y*-axis. The curve analysis showed that the radiomic model provides more benefit in distinguishing HCC from ICCA.

**Table 1:** Radiomic features in the radiomic analysis.

Types	Feature
Shape (*n* = 13)	Maximum3DDiameter, Maximum2DDiameterSlice, SphericityMinorAxis, Elongation, SurfaceVolumeRatio, Volume, MajorAxis, SurfaceArea, Flatness, LeastAxis, Maximum2D DiameterColumn, and Maximum2DDiameterRow
First-order statistics (*n* = 18)	InterquartileRange, Skewness, Uniformity, Median, Energy, RobustMeanAbsoluteDeviation, MeanAbsoluteDeviation, TotalEnergy, Maximum, RootMeanSquared, 90Percentile, Minimum, Entropy Range, Variance, 10Percentile, Kurtosis, and Mean
Textural features (*n* = 74) GLDM (*n* = 14)	GrayLevelVariance, HighGrayLevelEmphasis, DependenceEntropy, DependenceNonUniformity, GrayLevelNonUniformity, SmallDependenceEmphasis, SmallDependenceHighGrayLevelEmphasis, DependenceNonUniformityNormalized, LargeDependenceEmphasis, LargeDependenceLowGrayLevelEmphasis, DependenceVariance, LargeDependenceHighGrayLevelEmphasis, SmallDependenceLowGrayLevelEmphasis, and LowGrayLevelEmphasis
GLCM (*n* = 23)	JointAverage, SumAverage, JointEntropy, ClusterShade, MaximumProbability, Idmn, JointEnergy, Contrast, DifferenceEntropy, InverseVariance, DifferenceVariance, Idn, Idm, Correlation, Autocorrelation, SumEntropy, SumSquares, ClusterProminence, Imc2, Imc1, DifferenceAverageId, and ClusterTendency
GLRLM (*n* = 16)	ShortRunLowGrayLevelEmphasis, GrayLevelVariance, LowGrayLevelRunEmphasis, GrayLevelNonUniformityNormalized, RunVariance, GrayLevelNonUniformity, LongRunEmphasis, ShortRunHighGrayLevelEmphasis, RunLengthNonUniformity, ShortRunEmphasis, LongRunHighGrayLevelEmphasis, RunPercentage, LongRunLowGrayLevelEmphasis, RunEntropy, HighGrayLevelRunEmphasis, RunLengthNonUniformityNormalizedGrayLevelVariance, ZoneVariance, GrayLevelNonUniformityNormalized, and SizeZoneNon
GLSZM (*n* = 16)	UniformityNormalized, SizeZoneNonUniformity, GrayLevelNonUniformity, LargeAreaEmphasis, SmallAreaHighGrayLevelEmphasis, ZonePercentage, LargeAreaLowGrayLevelEmphasis, LargeAreaHighGrayLevelEmphasis, HighGrayLevelZoneEmphasis, SmallAreaEmphasis, LowGrayLevelZoneEmphasis, and ZoneEntropySmallAreaLowGrayLevelEmphasis
NGTDM (*n* = 5)	Coarseness, Complexity, Strength, Contrast, and Busyness
Wavelet transforms (*n* = 736)	Wavelet-HLL, wavelet-LHL, wavelet-LHH, wavelet-LLH, wavelet-HLH, wavelet-HHH, wavelet-HHL, and wavelet-LLL

GLCM: gray level cooccurrence matrix; GLRLM: gray level run length matrix; GLSZM: gray level size zone matrix; L: low; H: high.

The article "Classification of Hepatocellular Carcinoma and Intrahepatic Cholangiocarcinoma Based on Radiomic Analysis" was published in 2022. Journal: Comput Math Methods Med.

**Table 2:** Characteristics and clinical factors of patients.

Parameter	Training (*n* = 122)	Validation (*n* = 89)	*P* value
Sex			0.214
Men	93	61	
Women	29	28	
Age			0.441
<60	62	50	
≥60	60	39	
CT-evaluated results			0.246
HCC	108	83	
ICCA	14	6	
Laboratory findings			
AST	56.04 ± 52.66	64.15 ± 57.48	0.289
ALT	54.69 ± 49.81	65.31 ± 54.42	0.143
GGT	70.53 ± 41.55	73.69 ± 52.31	0.626
Total bilirubin	19.8 ± 23.24	17.6 ± 26.24	0.521
Platelet count	189.42 ± 63.24	181.89 ± 76.35	0.435
INR	1.06 ± 0.178	1.09 ± 0.193	0.245
AFP			0.251
>10	92	73	
≤10	30	16	
CEA			0.523
>5	8	4	
≤5	114	85	
CA199			0.976
>39	29	21	
≤39	93	68	
Histologic results			0.597
HCC	93	65	
ICCA	29	24	

HCC: hepatocellular carcinoma; ICCA: intrahepatic cholangiocarcinoma.

**Table 3:** The summary of model.

	Training			Validation		
	Radiomics	Evaluation	Radiomics vs evaluation	Radiomics	Evaluation	Radiomics vs evaluation
AUC	0.855	0.689	DeLong test = 0.01727	0.847	0.659	DeLong test = 0.01186
CI	(0.769, 0.942)	(0.591, 0.787)		(0.75, 0.945)	(0.545, 0.773)	
Cutoff	-0.9982626	1		-0.9960851	1	
Se	0.8275862	0.688172		0.8333333	0.6923077	
Sp	0.8602151	0.6896552		0.8307692	0.625	
PPV	0.6486486	0.8767123		0.6451613	0.8333333	
NPV	0.9411765	0.4081633		0.9310345	0.4285714	
DLR.Positive	5.9204244	2.2174432		4.9242424	1.8461538	
DLR.Negative	0.200431	0.4521505		0.2006173	0.4923077	
FP	13	9		11	9	
FN	5	29		4	20	

CI: 95% confidence interval.

The article "Classification of Hepatocellular Carcinoma and Intrahepatic Cholangiocarcinoma Based on Radiomic Analysis" was published in 2022. Journal: Comput Math Methods Med.

## Data Availability

The datasets analyzed during the current study are available from the corresponding authors on reasonable request.
